The article "The Msx1 Homeoprotein Recruits G9a Methyltransferase to Repressed Target Genes in Myoblast Cells" was retracted in 2023. Reasons: duplicated images; original data or images not available; concerns about the images.

# The Msx1 Homeoprotein Recruits G9a Methyltransferase to Repressed Target Genes in Myoblast Cells

**DOI:** 10.1371/journal.pone.0037647

**Published:** 2012-05-22

**Authors:** Jingqiang Wang, Cory Abate-Shen

**Affiliations:** Departments of Urology and Pathology & Cell Biology and Herbert Irving Comprehensive Cancer Center, Columbia University College of Physicians and Surgeons, New York, New York, United States of America; University of Crete, Greece

## Abstract

Although the significance of lysine modifications of core histones for regulating gene expression is widely appreciated, the mechanisms by which these modifications are incorporated at specific regulatory elements during cellular differentiation remains largely unknown. In our previous studies, we have shown that in developing myoblasts the Msx1 homeoprotein represses gene expression by influencing the modification status of chromatin at its target genes. We now show that genomic binding by Msx1 promotes enrichment of the H3K9me2 mark on repressed target genes via recruitment of G9a histone methyltransferase, the enzyme responsible for catalyzing this histone mark. Interaction of Msx1 with G9a is mediated via the homeodomain and is required for transcriptional repression and regulation of cellular differentiation, as well as enrichment of the H3K9me2 mark in proximity to Msx1 binding sites on repressed target genes in myoblast cells as well as the developing limb. We propose that regulation of chromatin status by Msx1 recruitment of G9a and other histone modifying enzymes to regulatory regions of target genes represents an important means of regulating the gene expression during development.

## Introduction

Cellular differentiation during development involves the coordinated change in expression of many thousands of genes in appropriate spatial and temporal contexts. A principal mechanism by which this occurs is through modification of the core histones (H3, H4, H2A, and H2B) that comprise nucleosomes, which are the fundamental units of chromatin. There are at least 8 distinct types of histone modifications, of which the most critical for transcriptional repression is lysine methylation, the enzymatic transfer of one or more methyl groups from the donor *S*-Adenosylmethionine (SAM) onto the ε-nitrogen of lysine [1], [2]. Genome-wide mapping studies using ChIP-Chip and ChIP-Seq have shown that di-methylation of histone H3 at lysine 9 (H3K9me2) is widely found at repressed genes during development and in embryonic stem cells [3], [4] while perturbation of the H3K9me2 mark results in a profound change in the repression status [5], [6]. The relevant histone lysine methyltransferase enzyme is G9a, a member of the highly conserved SET domain family, which, as part of a complex containing GLP, is responsible for catalyzing the H3K9me2 mark [7]–[11]. Thus, mutant mice lacking G9a are seriously impaired in the H3K9me2 mark and display embryonic lethality reflecting the consequences of global perturbation of gene repression [12]. Notably, the H3K9me2 mark, which is associated with transcriptional repression (regulated inhibition of gene expression), is distinct from tri-methylation of H3K9, which is associated with transcriptional silencing (permanent inhibition of gene expression), and is mediated by another SET domain protein, Suv39H1 [10], [13]–[15].

The article "The Msx1 Homeoprotein Recruits G9a Methyltransferase to Repressed Target Genes in Myoblast Cells" was retracted in 2023. Reasons: duplicated images; original data or images not available; concerns about the images.

The homeoprotein family comprises one of the major classes of sequence-specific DNA binding proteins, which regulate gene expression and cellular differentiation during development. Among its members is the Msx1 homeoprotein, which is expressed in diverse spatial and temporal domains during development but restricted to cells that have not yet begun to differentiate [16], [17]. In the myogenic lineage, for example, Msx1 is expressed in myogenic precursors during development as well as in adult myogenic satellite cells (*i.e*., stem cells), but not in differentiated myotubes [18]–[20]. Forced expression of Msx1 in myoblast cells inhibits their differentiation [21], [22], which is mediated by the actions of Msx1 as a transcriptional repressor. In particular, Msx1 represses *MyoD*, which is a principal regulator of myogenic differentiation, by binding to a key regulatory element, the *Core Enhancer Region* (CER) [20], [22]–[25] that regulates the timing of *MyoD* expression *in vivo* [26].

Previously, we have shown that regulation of myoblast differentiation and repression of *MyoD* expression by Msx1 is correlated with increased repressor marks at the CER of *MyoD* [25], which include increased tri-methylation of H3K27 (H3K27me3) [23]. We now show that in myoblasts as well as the developing limb genomic binding by the Msx1 homeoprotein promotes enrichment of the H3K9me2 mark on repressed target genes via recruitment of the G9a histone methyltransferase, the enzyme responsible for catalyzing this histone mark [7]–[11]. Interaction of Msx1 with G9a is mediated via the homeodomain and is required for transcriptional repression and regulation of cellular differentiation, as well as enrichment of the H3K9me2 mark in proximity to Msx1 binding sites on repressed target genes. Based on our findings on the recruitment of the H3K9me2 mark, in conjunction with our recently published findings regarding the role of Msx1 in recruiting H3K27me3 to target genes [23], we describe four distinct categories of Msx1 target genes that are distinguished by differential recruitment of the relevant histone methyltransferases. Our findings suggest that an important means of regulating gene expression during development involves the differential recruitment of histone modifying enzymes to regulatory regions of target genes to influence chromatin status.

The article "The Msx1 Homeoprotein Recruits G9a Methyltransferase to Repressed Target Genes in Myoblast Cells" was retracted in 2023. Reasons: duplicated images; original data or images not available; concerns about the images.

## Results

### Msx1 is Associated with H3K9me2 and Binds to G9a

Following from our previous study showing that repression of *MyoD* by Msx1 is correlated with increased repressor marks at a key regulatory element, the CER [25] and associated with increased tri-methylation of H3K27 (H3K27me3) [23], we looked more generally at how Msx1 may influence the modification status of core histones on target genes in myoblast cells. We found that Msx1 associates specifically with H3K9me2 but not H3K9me3 in co-immunoprecipitation assays using proteins immunopurified from C2C12 cells (Figure 1A). Notably, the H3K9me2 mark, which is associated with repression, is distinct from tri-methylation of H3K9, which is associated with transcriptional silencing [10], [13]–[15].

**Figure 1:** Msx1 binds to G9a/GLP via the homeodomain and the C-terminal region. (A) Co-immunoprecipitation assays were done using C2C12 cell protein extracts expressing Flag-Msx1 and immunoprecipitated with anti-Flag followed by immunoblotting for the indicated histone marks. (B) 293T cells were transfected with the indicated expression plasmids. Proteins were immunoprecipitated with Flag antibodies and immunoblotted with anti-Flag or Anti-Myc, as indicated. (C) *(Left)* C2C12 cell protein extracts expressing Flag-Msx1 were immunoprecipitated with anti-Flag following by immunoblotting with antibodies to detect the indicated proteins. *(Right)* Limb extracts (11.5 *dpc*) expressing endogenous Msx1 were immunoprecipitated with anti-Msx1 antibody (4F11) following by immunoblotting with antibodies to detect the indicated proteins. (D) Truncated Msx1 proteins expressed in 293T cells were immunopurified with anti-Flag followed by immunoblotting to detect G9a. Shown is the quantitative analyses of G9a, normalize to G9a input and Msx1 input. In each immunoprecipitation assays, 1 mg of protein was used and input was 1% of the total protein. (E) Schematic representation of Msx1 and truncated derivatives showing a summary of data.

Considering that Msx1 is associated with H3K9me2, we next asked whether Msx1 interacts with G9a, which is the enzyme that is responsible for this methyl mark. We found that both exogenous Msx1 expressed in C2C12 myoblast cells and endogenous Msx1 expressed in the developing limb interacted strongly with G9a, regardless of whether co-immunoprecipitation assays were done using antibodies to pull down Msx1 or G9a (Figure 1B and 1C). Msx1 also associated with GLP (Figure 1C), which forms a complex with G9a, but it did not interact with Suv39H1 (Figure 1C), which is responsible for tri-methylation of H3K9 and associated with gene silencing rather than repression [14].

The article "The Msx1 Homeoprotein Recruits G9a Methyltransferase to Repressed Target Genes in Myoblast Cells" was retracted in 2023. Reasons: duplicated images; original data or images not available; concerns about the images.

Msx1 has multiple functional domains that mediate interactions with protein partners, DNA binding, transcriptional repression and/or sub-nuclear location [23]–[25]. Analyses of truncated Msx1 proteins lacking these various functional domains revealed that the homeodomain of Msx1 is the primary domain required for its interaction with G9a (Figure 1D and 1E). In particular, a truncated Msx1 protein lacking the homeodomain [Msx1(1–172)] did not interact with G9a, while various other truncated Msx1 proteins that contained the homeodomain but lacked for example domains required for repression Msx1(139–303); Msx1(1–239); and Msx1(1–271)] interacted with G9a, albeit with varying degrees of efficacy (Figure 1D and 1E). Notably the homeodomain is required for DNA binding by Msx1 but also mediates interactions of Msx1 with other protein partners [16], [20], [23], [27]. Taken together, these findings indicate that Msx1 associates with G9a histone methyltransferase via the homeodomain, although the important caveat to these studies in the possible influence of these altered domains on the structure of the protein overall.

### Msx1 Genomic Binding Associates with Enrichment of the H3K9me2 Repressive Mark

Having established that Msx1 interacts with G9a, we next asked whether genomic binding by Msx1 is associated with increased levels of H3K9me2 on its repressed target genes in myoblast cells. In particular, we examined the status of H3K9me2 as a consequence of Msx1 expression at several sites on *MyoD* as well as several other myogenic regulators that are repressed by Msx1 [23], namely *Myf5*, *Angpt1*, *Myc*, *Six1,* and *Snai2* [28]–[34] (Figure 2A and 2B). Interestingly, we found that binding by Msx1 resulted in increased levels of H3K9me2 on certain but not all of these genomic binding sites. For example, Msx1 binding was associated with increased H3K9me2 on the CER regions of *MyoD* (MyoD-4; *P* = 4.4×10^−5^) and the −58 kb site of *Myf5* (Myf5-2; *P* = 2.4×10^−7^), both of which are known homeoprotein regulatory elements that control expression of these respective genes *in vivo* [26], [33], [34]. In contrast, H3K9me2 was not increased at the Msx1 binding sites of other target genes, such as *Snai2* (Figure 2B). Interestingly, for the target gene, *Six1*, where Msx1 binds to two sites (Six1–3 and Six1–6), only one of the sites (Six1–6) was enriched for H3K9me2 (Figure 2B); notably, we have found that the other site (Six1–3) displays an Msx1-dependent enrichment for an alternative methyl mark, H3K27me3 [23]. Furthermore, the Msx1-dependent enrichment of H3K9me2 was well correlated with recruitment of G9a binding to these sites (Figure 2C). In particular, ChIP-qPCR analyses revealed that G9a binding was significantly enriched at relevant Msx1 binding sites, including the CER (MyoD-4; *P = *0.001) and the −58 kb site of *Myf5* (Myf5-2; *P = *5.8×10^−5^), but not on its binding site on *Snai2,* which is also not enriched for H3K9me2 (Figure 2C, compare with Figure 2B). In the case of *Six1*, G9a was bound at only at the Msx1 site that was enriched for H3K9me2 (Six1–6; Figure 2B).

The article "The Msx1 Homeoprotein Recruits G9a Methyltransferase to Repressed Target Genes in Myoblast Cells" was retracted in 2023. Reasons: duplicated images; original data or images not available; concerns about the images.

**Figure 2:** Msx1 genomic binding associates with enrichment of the H3K9me2 repressive mark in myoblast cells. (A) Diagram of six Msx1 repressed target genes [23] showing the positions of Msx1 binding sites and known regulatory regions as well as their overlap; also shown is a negative control site. DRR: Distal Regulatory Region. (B) ChIP-qPCR analyses showing the relative levels of H3K9me2 at Msx1 genomic binding sites in C2C12 cells. ChIP data are expressed as relative enrichment of H3K9me2 normalized to input in C2C12 cells expressing or lacking Msx1. *(Inset)* ChIP data expressed as fold enrichment of H3K9me2 in C2C12 cells expressing Msx1 versus the control cells lacking Msx1 (and normalized to input). (C) ChIP-qPCR assays were done using C2C12 cells expressing Flag-Msx1 or a control vector to evaluate binding of G9a to the indicated Msx1 target sequences. ChIP data are expressed as relative enrichment of G9a binding normalized to input in C2C12 cells expressing or lacking Msx1. *(Inset)* ChIP data are expressed as fold enrichment of G9a binding in C2C12 cells expressing Msx1 versus the control cells lacking Msx1 (and normalized to input). In B and C, the * indicate the following: ***P<0.0001, **P<0.001, *P<0.01.

To investigate whether these findings were also relevant for endogenous Msx1 *in vivo*, we performed ChIP analysis using limb from wild-type or *Msx* mutant embryos. We found that the levels of H3K9me2 were significantly reduced in the *Msx* mutant versus wild-type limb at the MyoD CER (MyoD-4; *P* = 1.7×10^−5^) and the −58 kb region of *Myf5* (Myf5-2; *P* = 4.9×10^−5^) but not at Snai2-1 (Figure 3). Notably, similar to our findings in the myoblast cells, levels of H3K9me2 on the *Six1* gene were significantly reduced in the *Msx* mutant versus wild-type limb at the Six1–6, but not at Six1–3 (Figure 3). Taken together, these data suggest that, for the endogenous protein *in vivo* as well as the exogenous protein in myoblast cells, Msx1 recruits G9a to selected genomic targets where it promotes enrichment of the H3K9me2 repressive mark in the vicinity of its binding.

The article "The Msx1 Homeoprotein Recruits G9a Methyltransferase to Repressed Target Genes in Myoblast Cells" was retracted in 2023. Reasons: duplicated images; original data or images not available; concerns about the images.

**Figure 3:** Msx1 genomic binding associated with enrichment of the H3K9me2 repressive mark in the developing limb. ChIP-qPCR analyses show relative levels of H3K9me2 at Msx1 genomic binding sites in *Msx1; Msx2* conditional mutant versus wild-type limb (13.5 *dpc*). ChIP data are expressed as relative enrichment of the H3K9me2 mark normalized to input. *(inset)* ChIP data expressed as fold enrichment in wild-type embryonic limb versus *Msx1*; *Msx2* conditional mutant embryonic limb (and normalized to input). The * indicate the following: ***P<0.0001, **P<0.001, *P<0.01.

### Association of Msx1 with G9a is Required for Regulation of Myoblast Differentiation

We next investigated the consequences of Msx1 association with G9a for regulation of myogenic differentiation by evaluating the consequences of G9a knock-down in C2C12 myoblast cells. We used two independent G9a siRNAs and verified their efficacy and specificity in C2C12 cells using q-PCR to evaluate G9a mRNA levels and Western blotting to detect levels of G9a protein or levels of histone marks (Figure 4A-C); for most assays, only one siRNA is shown. The consequences of G9a knock-down for regulation of differentiation by Msx1 were evaluated by the appearance of myotubes and by Western blot detection of markers of terminal muscle differentiation, namely myosin heavy chain (MHC) and Myogenin (Figure 4D and 4E). Without exogenous Msx1 expression, C2C12 cells (Vector) were differentiated by 3 days after induction regardless of whether they expressed the control or G9a siRNA as evident by myotubes formation (Figure 4D, top panel) and expression of MHC and Myogenin (Figure 4E, left panel). However, as we have shown previously [21], [24], [25], Msx1 completely abrogates differentiation of C2C12 cells, as evident by the absence of myotubes (Figure 4D, left bottom panel) and lack of expression of MHC and Myogenin (Figure 4E, right panel). In contrast, depletion of G9a reverted these inhibitory effects of Msx1 on myoblast differentiation, as evident from the appearance of myotubes (Figure 4D, right bottom panel) and expression of MHC and Myogenin (Figure 4E, right panel).

**Figure 4:** Association of Msx1 with G9a is required for regulation of myoblast differentiation. (A) Quantitative PCR to determine the level of G9a mRNA following knock-down by siRNA, mRNAs were prepared 48 hours after transfection with the indicated siRNA. (B) Western blot assay for efficiency of G9a knock-down, C2C12 cells were transfected with the indicated siRNA, extracts prepared 72 hours after transfection and analyzed by western blotting for the indicated proteins. (C) Western blot assay for histone marks. C2C12 cells were transfected with the indicated siRNA, extracts prepared 72 hours after transfection and analyzed by western blotting for the indicated histone marks. (D) Differentiation assay of C2C12 cells expressing (+) or lacking (-) Msx1 along with the control or G9a siRNA. Micrographs of C2C12 cells show the absence of myotubes in Msx1-expressing cells but not in cells also expressing the G9a siRNA on Day 3 after differentiation. (E) Western blots analyses of markers of terminal muscle differentiation, MHC and Myogenin on Day 3 after differentiation. (F) Immunofluorescence assays done on Day 2 after differentiation as detected using antibody for MHC and the nuclear marker TOPRO3. The scale bars represent 50 µm. (G) Quantitative analyses of myogenic index on Day 2 after differentiation. The percentage of MHC+ cells in vector cells with control siRNA was given a value of 100%. In A and G, the * indicate the following: ***P<0.0001, **P<0.001, *P<0.01.

The article "The Msx1 Homeoprotein Recruits G9a Methyltransferase to Repressed Target Genes in Myoblast Cells" was retracted in 2023. Reasons: duplicated images; original data or images not available; concerns about the images.

We quantified the differentiation status of the C2C12 cells at 2 days after induction of differentiation using an antibody for MHC to detect the MHC+ cells and determine the myogenic index [35]. In vector cells, depletion of G9a resulted in a higher myogenic differentiation compared with those expressing the control siRNA (Figure 4F and 4G), consistent with a role G9a in myogenic differentiation as reported recently [35]. However, in Msx1-expressing cells, depletion of G9a restored the myogenic differentiation nearly the levels without Msx1 (Figure 4F and 4G). These findings demonstrate that G9a is essential for Msx1 to inhibit myogenic differentiation in these myoblast cells.

### Association of Msx1 with G9a is Required for Transcriptional Repression

We next investigated the consequences of Msx1 association with G9a for transcriptional repression following knock-down of G9a in C2C12 myoblast cells. Depletion of G9a significantly reduced Msx1 binding to genomic sites of repressed genes in myoblast cells in ChIP assays, as exemplified for the CER (MyoD-4; *P* = 1.1×10^−7^) and the −58 kb element of *Myf5* (Myf5-2; *P* = 3.8×10^−4^) (Figure 5A). Interestingly however, analyses of Msx1 binding *in vitro* in gel shift assays showed that G9a knock-down did not inhibit binding by Msx1 to these genomic target sequences, namely the MyoD CER (MyoD-4) or Myf5-1 (Figure 5B). Notably, we have previously shown a distinction between binding of Msx1 *in vitro* and its ability to bind with target sequences *in vivo*, which is dependent on interactions with its protein partners *in vivo* [23], [24]. Thus, while G9a may not directly affect the affinity of Msx1 for its binding sites (Figure 5B), considering that depletion of G9a impaired in Msx1 ability to interact with genomic binding sites *in vivo* (Figure 5A), G9a may affect the ability of Msx1 to access authentic target sites in myoblast cells.

The article "The Msx1 Homeoprotein Recruits G9a Methyltransferase to Repressed Target Genes in Myoblast Cells" was retracted in 2023. Reasons: duplicated images; original data or images not available; concerns about the images.

**Figure 5:** Association of Msx1 with G9a is required for transcriptional repression. (A) ChIP-qPCR analyses showing relative Msx1 binding in C2C12 cells expressing or lacking Msx1 as well as a control or G9a siRNA. ChIP data are expressed as fold enrichment of Msx1 binding in C2C12 cells expressing Msx1 versus control cells lacking Msx1. (B) Gel shift analyses were done using nuclear extracts from C2C12 cells expressing Flag-Msx1 as well as the control or G9a siRNA with DNA sequences corresponding to the MyoD CER (MyoD-4) and Myf5-1. The * indicate the protein-DNA binding bands, the arrowhead indicates the free probes. (C) Expression levels of Msx1 target genes in Msx1-expressing or lacking Msx1 C2C12 cells also expressing the control or G9a siRNA. Data are expressed as the fold change of mRNA relative to that of the control siRNA cells. The * indicate the following: ***P<0.0001, **P<0.001, *P<0.01. (D) Western blots analyses showing levels of MyoD and Myf5 protein following by G9a knock-down in Msx1-expressing or lacking Msx1 C2C12 cells.

Notably, the diminished binding of Msx1 to repressed genes in myoblast cells as a consequence of G9a knock-down was accompanied by a partial abrogation of repression of its target genes, including *MyoD, Angpt1*, *Myc* and *Six1* following knock-down of G9a in Msx1-expressing but not the cells without Msx1 (Vector) (Figure 5C and 5D). The notable exception was *Myf5*, which was increased in expression at the protein and mRNA levels in the vector cells (lacking exogenous Msx1) following G9a knock-down (Figure 5C and 5D). Although depletion of G9a in C2C12 cells does not affect MyoD mRNA and protein levels (see Figure 5C and 5D), it may inhibit its transcriptional activity, in turn leading to up-regulation of *Myf5* (Figure 5C and 5D, top panel), which is consistent with a recent study showing that G9a interacts with MyoD to constrain its transcriptional activity [35]. Finally, following G9a knock-down in Msx1 expressing C2C12 cells, we observed a significant reduction in the H3K9me2 mark, but not the H3K9me3 mark, on Msx1 target genomic binding sites such as CER (MyoD-4; *P* = 7.8×10^−5^) and the −58 kb region of *Myf5* (Myf5-2, *P* = 4.2×10^−4^), as well as on the genes that are regulated by G9a but not Msx1 such as *MageA2*, *Major satellite*, and *Wfdc15a*, but not on a gene (*GAPDH*) that is not regulated by either Msx1 or G9a (Figure 6A–H) [6], [12]. Taken together, these findings demonstrate that the interaction of Msx1 with G9a in myoblast cells is essential for Msx1 to bind and repress target genes in cells and for enrichment of the H3K9me2 repressive mark at specific genomic binding sites.

The article "The Msx1 Homeoprotein Recruits G9a Methyltransferase to Repressed Target Genes in Myoblast Cells" was retracted in 2023. Reasons: duplicated images; original data or images not available; concerns about the images.

**Figure 6:** Binding analyses of H3K9 methyl marks in G9a knock-down cells. ChIP-qPCR assays were done using C2C12 cells expressing Flag-Msx1 as well as the control or G9a siRNA using anti-H3K9me2 or anti-H3K9me3 or control IgG, as indicated. ChIP data are expressed as relative enrichment normalized to input in control siRNA cells or G9a knock-down cells.

### The G9a associated with Redistribution of H3K27me3 by Msx1 to Genomic Sites

Finally, since we have shown previously that repression by Msx1 is correlated with increased tri-methylation of H3K27 (H3K27me3) [23], we asked whether Msx1 association with G9a affected the H3K27me3 mark on target genes. Since depletion of G9a did not reduce the total level of H3K27me3 (Figure 4C), we asked whether Msx1 association with G9a is required for the Msx1-dependent redistribution of H3K27me3 on its genomic bound sites. In the presence of control siRNA, Msx1 promotes enrichment of the H3K27me3 repressive mark on its genomic sites, such as *MyoD-2, MyoD-4, Myf5-1* and *Myf5*-2 [23] (Figure 7A). In contrast, genes that were neither bound nor regulated by Msx1, such as *Dkk1, En2,* and *Irx1* had *reduced* levels of H3K27me3 in Msx1-expressing C2C12 cells with control siRNA [23] (Figure 7B). However in Msx1 expressing C2C12 cells, knock-down of G9a dramatically reduced the H3K27me3 mark on Msx1 genomic sites (Figure 7A), while it resulted in reversed the H3K27me3 reduction at *Dkk1, En2,* and *Irx1* associated with exogenous Msx1 expression (Figure 7B). Furthermore, since the association of Msx1 with the nuclear periphery is associated with the redistribution of the H3K27me3 mark [23], we asked whether G9a affects the sub-nuclear location of Msx1. Strikingly, we found that depletion of G9a dramatically interrupted Msx1 nuclear periphery localization (Figure 7C). These findings suggest that Msx1 association with G9a contributes to the Msx1-dependent redistribution of H3K27me3 genomic bound sites by affecting the nuclear periphery localization of Msx1.

**Figure 7:** G9a is required for Msx1-induced redistribution of H3K27me3 by Msx1 and localization of Msx1 at the nuclear periphery in C2C12 myoblasts. (A) ChIP-qPCR analyses of H3K27me3 mark on Msx1 target genes in C2C12 cells lacking Msx1 or expressing exogenous Msx1 also expressing the control or G9a siRNA. ChIP data are expressed as relative enrichment of the H3K27me3 mark normalized to input. (B) ChIP-qPCR analyses of H3K27me3 mark on genes not bound by Msx1 in C2C12 cells lacking Msx1 or expressing exogenous Msx1 also expressing the control or G9a siRNA. ChIP data are expressed as relative enrichment of the H3K27me3 mark normalized to input. (C) Immunofluorescence assays were done on C2C12 cells expressing exogenous Msx1 together with the G9a siRNA or a control siRNA and detected using antibodies for Msx1 or by detection of the nuclear marker TOPRO3. Quantitative analyses of nuclear localization for Msx1 using ImageJ show representative data from 3 independent assays, each counting a minimum of 20 cells per variable. The scale bars represent 5 µm.

The article "The Msx1 Homeoprotein Recruits G9a Methyltransferase to Repressed Target Genes in Myoblast Cells" was retracted in 2023. Reasons: duplicated images; original data or images not available; concerns about the images.

## Discussion

The impact of Msx1 on cellular differentiation during development is dependent on its ability to repress the expression of regulatory genes in specific cellular contexts, such as occurs for *MyoD* in cells of the myogenic lineage [22], [24], [25]. Our current findings suggest that these activities of Msx1 are mediated by its ability to directly influence the methylation status of nucleosomes on selected regulatory elements to which it is bound in myoblast cells (Figure 8). Our findings further indicate that this reflects, in part, recruitment of the G9a histone methyltransferase to these regulatory sites, which in turn promotes methylation of core histones in the vicinity of Msx1 binding (Figure 8; Table S1). Notably, recruitment of the G9a histone methyltransferase by Msx1 is mediated via the homeodomain, which is the defining feature of this family of sequence specific developmental regulators [16], [20], [22], [24], [25]. Implicit in this observation is that other homeoproteins may also recruit methyltransferase enzymes to target genes as a means of regulating their expression.

**Figure 8:** Working model. As described in the text, we have proposed that binding of the Msx1 homeoprotein to specific target genes brings G9a and/or Ezh2 to the regulatory regions of these genes to influence histone modifications. According G9a and Ezh2 bound status, the Msx1 bound and down-regulated target genes were categorized in 4 categories. (A) Category I, Msx1 brings G9a and Ezh2 to the same site on target genes. (B) Category II, Msx1 brings G9a and Ezh2 to the same target genes but at different sites. (C) Category III, Msx1 only brings Ezh2 to the Msx1 bound site on target genes. (D) Category IV, Msx1 do not brings ether G9a or Ezh2 to the target genes, but Msx1 may brings other factors to Msx1 bound site to repress target genes expression.

However, G9a is not recruited to all Msx1 target genes. Moreover, Msx1 also interacts via the homeodomain with another histone methyltransferase, Ezh2, which leads to enrichment of its respective histone mark, namely H3K27me3, on certain target genes (Figure 8; Table S1) [23]. In fact, we can identify 4 scenarios in which Msx1 differentially recruits histone methyltransferases to target genes to regulate their expression. In particular, in the first case Msx1 recruits both H3K9me2 and H3K27me3 repressive marks at the same binding site, as is the case for target genes, such as, *MyoD*, *Myf5*, *Myc*, and *Angpt1* [18], [26], [28], [31], [33], [34]. In the second scenario, Msx1 recruits both H3K9me2 and H3K27me3 repressive marks to target genes, but at the different sites. For instance, Msx1 binds to two sites on *Six1* (Six1–3 and Six1–6), one of the sites (Six1–6) is enriched for H3K9me2 while the other site (Six1–3) displays an Msx1-dependent enrichment for H3K27me3 [23], [29], [30]. In the third case, Msx1 only recruits the H3K27me3 mark, as in the case for *Snai2*, *Met*, and *Id3* [32], [36], [37]. The final case is target genes that are bound by Msx1, but are not enriched for either H3K9me2 or H3K27me3, such as *Clcn3* and *Fgf7* [38], [39].

The article "The Msx1 Homeoprotein Recruits G9a Methyltransferase to Repressed Target Genes in Myoblast Cells" was retracted in 2023. Reasons: duplicated images; original data or images not available; concerns about the images.

Implicit in this description is the important but yet unanswered question regarding how Msx1 recruits multiple histone methyltransferases to distinct target genes in specific spatial contexts. Therefore, Msx1 may interact with multiple histone methyltransferases to influence the expression of target gene in dynamic spatial contexts. Furthermore, since the region of methyltransferases recruitment is the homeodomain, a conserved motif, our findings raise the possibility that other homeoproteins may also function by promoting the recruitment of histone modifying enzymes to target genes. Thus, our findings demonstrate a novel means by which homeoproteins can regulate gene expression during development by interacting with histone modifying enzymes to directly influence the chromatin status of target genes.

## Materials and Methods

### Plasmids

Most of the expression plasmids used in this study has been described previously [24], [25]. As indicated, pcDNA3 expression plasmids were used for transient transfection and pLZRS-IRES-GFP plasmids for retroviral gene transfer. Flag-tagged G9a was generated using PCR amplification and cloned into BamH I – Xho I sites of pcDNA3. The complete sequences of all PCR-amplified constructs were confirmed.

### Cell Culture Analyses

Cell culture studies were done using human 293T cells (ATCC) or mouse C2C12 myoblast cells (ATCC). Cells were maintained in DMEM supplemented with 10% fetal bovine serum in humidified atmosphere with 5% CO2 at 37C. For myoblast differentiation assays, undifferentiated C2C12 cells were grown in media containing 10% fetal bovine serum, and differentiation was induced by shifting cells to media containing 2% horse serum 21,24,25. Transient transfection was performed using Lipofectamine 2000 reagent (Invitrogen). For retroviral gene transfer, replication-defective retroviruses were made in ecotropic Phoenix retroviral packaging cells (ATCC) by transfection of the relevant pLZRS-IRES-GFP plasmid derivatives using Lipofectamine 2000 reagent (Invitrogen). C2C12 myoblast cells were seeded 1 day before infection and infected with viral supernatants for two consecutive days. For siRNA, C2C12 cells were first infected with viruses expressing Msx1 or the empty vector and then transfected with siRNA against G9a (Ambion) using the Lipofectamine RNAiMAX reagent (Invitrogen) according to the manufacturer’s recommendations. For the control siRNA using *Silencer*® Select negative control #1 siRNA (Ambion). The sequences of G9a siRNA (Ambion) used in these studies are provided in Table S2. Quantitative analyses of differentiation of the G9a knock-down C2C12 cells were done by immunofluorescence staining with MHC antibody (see the below). Quantitative analyses of myogenic index were preformed on Day 2 after differentiation. Myogenic index calculation was done as described in [35]. At least 3 independent assays were done per variable, counting a minimum of 500 cells per variable for each independent assay. The percentage of MHC+ cells in vector cells with control siRNA was given a value of 100%.

The article "The Msx1 Homeoprotein Recruits G9a Methyltransferase to Repressed Target Genes in Myoblast Cells" was retracted in 2023. Reasons: duplicated images; original data or images not available; concerns about the images.

### Analyses of *Msx1* Mutant Embryos

All experiments using animals were performed according to protocols approved by the Institutional Animal Care and Use Committee at Columbia University Medical Center. The *Msx1* mutant were performed using a compound *Msx1; Msx2* conditional allele [40] crossed to a ubiquitously-expressed tamoxifen-inducible Rosa26^CreERT2^ allele [41] to generate mice of the genotype *Rosa26^CreERT2/+^*; *Msx1^lox/lox^; Msx2^lox/lox^*. Targeted deletion was induced by delivery of tamoxifen in corn oil (2 mg/40 grams; Sigma-Aldrich) by oral gavage at embryonic day 9.5 (9.5 *days post-coitum, dpc*); targeted deletion in the tissue of interest (*i.e.,* the limb) was confirmed by PCR analyses. The analyses described herein focused on mid-gestation embryos, from days 10.5 to 13.5 *dpc*, at which developmental stages the limb buds are maturing and *Msx1* expression is robust in the limb mesenchyme [16], [42]. Embryos were collected from timed mating with noon on the day of the plug considered to be embryonic day 0.5; embryos were genotyped from yolk sac DNA. For ChIP assays, freshly dissected limbs were collected in PBS with protease inhibitor cocktail and disrupted using a Polytron homogenizer. Tissue extracts were cross-linked with 1% formaldehyde for 30 minutes at room temperature, cross-linking was stopped with 0.1 M Glycine, and cross-linked limb was collected by centrifugation and processed for ChIP-qPCR analyses as below.

The article "The Msx1 Homeoprotein Recruits G9a Methyltransferase to Repressed Target Genes in Myoblast Cells" was retracted in 2023. Reasons: duplicated images; original data or images not available; concerns about the images.

### Real-time PCR for Gene Expression

Real-time PCR was done using RNA isolated from C2C12 cells, using Trizol reagent (Invitrogen), and purified using an RNeasy kit (Qiagen). First strand cDNA was synthesized using SuperScript III kit (Invitrogen) and quantitative real-time PCR was performed using SYBR green reagent (Qiagen) in the Realplex^2^ machine (Eppendorf). Expression values were normalized to *GAPDH*. At least three independent experiments were performed for each gene. The average values are given as the mean ± SD. The primer sequences for real-time PCR using in this study were provided in Table S2.

### Chromatin Immunoprecipitation (ChIP)

ChIP analysis was performed as described previously [24], [25]. Briefly, C2C12 cells expressing or lacking Msx1 and/or siRNA for G9a were cross-linked using 1% formaldehyde and genomic DNA was sonicated and then the relevant protein-DNA complexes were isolated by immunoprecipitation. ChIP analysis from limb, the cross-linked limb tissue was sonicated and then the relevant protein-DNA complexes were isolated by immunoprecipitation. The antibodies were used for ChIP assays were provided in Table S3. Quantitative real-time PCR was performed in triplicate using SYBR green reagent (Qiagen) using a Realplex^2^ machine (Eppendorf). At least three independent experiments were done for each assay. Primer sequences for ChIP-qPCR analyses were provide in Table S2.

### Immunoprecipitation and Western Blotting Analyses

For Western blotting, C2C12 cells were lysed in RIPA buffer and proteins were analyzed using ECL plus Western Blotting Detection (GE Healthcare) by indicated antibodies (Table S3). For immunoprecipitation assays, C2C12 cells were lysed in RIPA buffer and proteins were immunoprecipitated by addition of antibodies [24], [25]. Where indicated, nuclear extracts from embryonic limbs were obtained by homogenization in hypotonic buffer (20 mM HEPES [pH 7.4], 5 mM NaCl, 1 mM EDTA, 10 mM MgCl_2_, 1 mM DTT, and protease inhibitor cocktail) to isolate nuclei followed by extraction of nuclear proteins in buffer BC1000 (25 mM HEPES [pH 7.9], 10% glycerol, 0.2 mM EDTA, 1000 mM KCl, protease inhibitor cocktail, and PMSF) containing 0.1% NP40. The samples were then sonicated, centrifuged at 16,000 g, and then dialyzed against BC200 (25 mM HEPES [pH 7.9], 10% glycerol, 0.2 mM EDTA, 200 mM KCl, protease inhibitor cocktail, and PMSF) containing 0.1% NP40. Immunoprecipitations were done in BC200 containing 0.1% NP40 and immunoprecipitated proteins were analyzed using ECL plus Western Blotting Detection (GE Healthcare). The antibodies were used for immunoprecipitation and immunoprecipitation Western blotting were provided in Table S3.

The article "The Msx1 Homeoprotein Recruits G9a Methyltransferase to Repressed Target Genes in Myoblast Cells" was retracted in 2023. Reasons: duplicated images; original data or images not available; concerns about the images.

### Gel Shift Assay

The probe of MyoD CER (MyoD-4) and Myf5-1 were generated fragment from ChIP DNA by using PCR method with ChIP-qPCR primer sets (Table S2). For nuclear extracts, the C2C12 cells were homogenized in hypotonic buffer. The nuclei were incubated for 10 min on ice and then pelleted by centrifugation at 8,000 g, and resuspended in BC1000 buffer containing 0.1% NP40 to extract nuclear proteins. The samples were then sonicated, centrifuged at 16,000 g, and dialyzed against BC200 containing 0.1% NP40. The binding reaction was perform in 1× binding buffer (10 mM Tris-HCl pH 7.5, 5 mM NaCl, 0.7 mM MgCl_2_, 0.1 mM EDTA, 5% Glycerol, 0.05% NP-40, and 50 µg/ml BSA, 2.5 mM DTT) with 2 µg poly d(I-C), 50 ng probe, and 5 µg of nuclear protein from C2C12 cells expressing Flag-Msx1 as well as the control or G9a siRNA in total volume of 20 µl. Binding was done at room temperate for 20 min. Protein-DNA binding complexes were resolved by electrophoresis. After finished running the gel, the gel was stained by SYBR Safe DNA gel stain (Invitrogen) and the digital imagines were captured by CCD camera.

### Immunofluorescence Analyses

Immunofluorescence analyses were done as described previously [23]. Briefly C2C12 cells seeded on 1-well BD Falcon™ CultureSlide and transfected with the indicated Msx1 plasmids and, where indicated, also with the siRNA for G9a. Cells were fixed in 4% PFA in PBS with 1% sucrose and permeabilized by incubation in an isotonic solution, 0.5% Triton X-100 (10% sucrose, 50 mM NaCl, 6 mM MgCl_2_, 20 mM HEPES [pH 7.2], 0.5% Triton X-100). After blocking with 1% BSA (bovine serum albumin) in PBS, cells were incubated for 1.5 hours at room temperature with primary antibodies. Following incubation with primary antibodies, samples were washed in PBS containing 0.1% Tween 20 followed by incubation for 1 hour with TOPRO 3 and AlexaFluor 488 and/or AlexaFluor 555 secondary antibodies (Molecular Probes). Immunofluorescence staining was visualized using a Leica TCS SP5 inverted confocal microscope equipped with argon/krypton and helium/neon lasers capable of excitation wavelengths 488, 555, and 642 nm. Details of primary antibodies are provided in Table S3. The Msx1 sub-nuclear localization was quantified using ImageJ (http://rsb.info.nih.gov/ij/) [43]. A line was drawn from the nuclear periphery to the nuclear center, and along this line, the fluorescence intensity was recorded; the pixel values versus radial position were used to generate the quantitative plot.

The article "The Msx1 Homeoprotein Recruits G9a Methyltransferase to Repressed Target Genes in Myoblast Cells" was retracted in 2023. Reasons: duplicated images; original data or images not available; concerns about the images.

### Statistical Analysis

At least three independent experiments were performed for each assay. The average values of the parallel experiments are given as the mean ± SD. Comparison of differences among the groups was carried out by Student’s *t*-test. Significance was defined as *p*<0.01. (***p<0.0001, **p<0.001, *p<0.01).

## Supporting Information

Table S1 **Summary of ChIP data for Msx1 bound and down-regulated target genes.**
(DOCX)

Table S2 **List of primers used for ChIP-qPCR, RT-PCR and RNA interference.**
(DOCX)

Table S3 **List of antibodies used in this study.**
(DOCX)
